The article "Post-COVID-19 investor psychology and individual investment decision: A moderating role of information availability" was retracted in 2025. Reasons: unreliable results or conclusions; a conflict of interest; concerns about the peer review; concerns about the citations.

# Post-COVID-19 investor psychology and individual investment decision: A moderating role of information availability

**DOI:** 10.3389/fpsyg.2022.846088

**Published:** 2022-09-28

**Authors:** Naveed Jan, Vipin Jain, Zeyun Li, Javeria Sattar, Korakod Tongkachok

**Affiliations:** ^1^Business School, Shandong Normal University, Jinan, China; ^2^Department of Management and Technology, Teerthanker Mahaveer University, Moradabad, Uttar Pradesh, India; ^3^School of Humanity, University Sains Malaysia, George Town, Malaysia; ^4^Lahore Business School, The University of Lahore, Lahore, Pakistan; ^5^Department of Law, School of Law, Thaksin University, Songkhla, Thailand

**Keywords:** psychological biases, investment decision, COVID-19, stock markets, China

## Abstract

This study aims to investigate the influence of psychological biases on the investment decision of Chinese individual investors after the pandemic of COVID-19 with a moderating role of information availability. A cross-sectional method with a quantitative research approach was employed to investigate the hypothesized relationships among variables. The snowball sampling technique was applied to collect the data through a survey questionnaire from individual investors investing in the Chinese stock market. Smart-PLS statistical software was used to analyze the data and for the estimation of hypotheses. Results indicated that overconfidence, representative bias, and anchoring bias have a significant and positive influence on investment decisions during the post-Covid-19 pandemic; however, the availability bias has insignificant and negative effects on the investment decision during the post-COVID-19 pandemic. Moreover, findings indicated that information availability has a significant moderating role in the relationship of psychological biases with the investment decision during the post-COVID-19 pandemic. This study contributes to the body of knowledge regarding behavior finance, psychological biases, and investment decision in emerging stock markets. The findings of the present study improve the understanding that how investors’ psychology affects their investment decisions.

## Introduction

At the start of January 2020, the spread of coronavirus (COVID-19) in China not only resulted in a huge loss of lives but also continued to influence the economy all over the globe negatively (Fernandez-Perez et al., 2021). All countries in the world responded differently to this pandemic. For instance, Sweden imposed very few social restrictions in this pandemic. In contrast, many other countries imposed strict restrictions, including complete lockdowns and social isolation. Similarly, stock markets all around the globe witnessed a varying level of decline in response to COVID-19, more than 30% in cases of some markets. Here, the question arises that what factors are responsible for varying responses of investors. In behavioral finance, investment behavior is recognized as an innovative research sub-area that deals with the ways investors perceive, forecast, examine and review the decision-making process that comprises investment psychology, gathering information, contextualizing, understanding, research, and investigation. The rationality of investors and market efficiency is considered as the main hypothesis by a majority of finance researchers in explaining financial concepts. Investors’ decisions are always assumed rational, and markets are considered to be lined up for perceived utility maximization. In contrast, numerous researchers in the last few decades indicated that traditional finance theories are not enough to describe the irrational behavior of investors while making decisions regarding investment (Huang et al., 2018). In a practical situation, investors are influenced by many behavioral biases that make their behavior irrational (Thaler and Ganser, 2015). In literature, various studies of behavioral finance examined and found that psychological elements of investors influence their investment decisions (Ahmed et al., 2020). In contrast to the traditional finance assumptions, which assume investors to be always rational, behavioral finance considers and theoretically proves that investors are always not rational but are irrational when deciding on an investment. Moreover, the recent global pandemic of COVID-19 discloses the significance of highlighting factors that influence the behavior of investors in evaluating the decision-making process while investing. Behavioral finance theory states that a deep understanding of behavioral psychology helps in the understanding of irregularities regarding the stock market and investment decisions. In addition, understanding the psychology of investors while deciding investment supports the investors in dealing with their behavioral biases and converting them to beneficial returns that urge them for further investment (Boda and Sunitha, 2018). The key objective of this study is to investigate and understand the investment behavior of an individual chronologically. In this study, the impact of psychological and emotional elements on market variations is incorporated with the emphasis on investor rationality in explaining the psychological effects of investing. Traditional finance perceives that investors are sensitive and typical in making investment decisions in the stock market, which is why they are not more involved in risk-return trade-offs and manipulating figures. The efficient market model states that investors should evaluate all the available relevant information and decide on investment impartially and without any biases. In contrast, psychologists recommended that individuals behave in irrational manners as opposed to the supposition of economists. Babajide and Adetiloye (2012) and Bashir et al. (2013) found that investors normally are not as rational as they are depicted. Hence, these irregularities in the behaviors of investors can be examined and explained by behavioral finance. Behavioral finance incorporates how individuals, groups of investors, experts, and portfolio managers are affected by psychological elements. It also attempts to comprehend how cognitive errors and emotions stimulate investors’ attitudes (Kengatharan and Kengatharan, 2014). Moreover, it also attempts to investigate why investors act in irrational manners and as opposed to perceived manners. In the literature of behavioral finance, researchers have highlighted several psychological factors that play a role in the decision-making of investors while investing in the stock market. The spread of COVID-19 particularly influenced every aspect of life by influencing public health. Various significant consequences are carried by the worldwide stock and financial market sustainability (Ali, 2020; Guo et al., 2020). Investors are also part of a social setup that is why their sentiments, emotions, optimism, and pessimism about upcoming stock prices are shaped accordingly. Stock prices of Shanghai, Nikkei’s, and Dow Jones witnessed a sharp decline in response to the volatile emotions of an investor during the period of COVID-19. This study focuses on the association between the sentiments of investors and stock prices. Additionally, Li et al. (2014) and Chen et al. (2014) elucidated that previous returns of the market are important determinants of investors sentiment; however, current market returns shape investor sentiment. A positive association between stock markets and sentiment points out that the sentiment of an investor is a contrarian predictor of upcoming market profits. Accordingly, there will be a strong impact on sentiments if stocks are easy or hard to evaluate and they are negatively or positively influenced by sentiments (Aissia, 2016; Xiang et al., 2021). Lan et al. (2020) evaluated the fundamental macroeconomic element with the help of market index return, and found that pre-communication of irregular returns came from sentiments of investors. Overvalued determined sentiments are modified within 1 month after their communication. In the meantime, the market timer deals with the situation and takes the benefit of delivering season stocks. In the high-sentiment period, stock price sensitivity is witnessed high in terms of the positive news regarding returns. On the other hand, stock price sensitivity is found low in the period of low sentiment. Literature suggests that general irregularity in stock prices are due to sentiments of investor because mispricing is derived from sentiments of earning (Mian and Sankaraguruswamy, 2012; Oprea and Brad, 2014; Zhang et al., 2019; Cheema et al., 2020). High completion in the market specifies that sentiments and market returns have a positive association, while this relation is negative in the case of low competition in the market. Though crises in the financial market change the condition regardless of the level of competition, still a positive association prevails between market returns and sentiments (Ryu et al., 2020). In comparison to a common person or layman, investors accept psychological stress more intensively and considerately. Irrespective of the spread of COVID-19, fear is communicated by social media rumors and news. Tetlock (2015) concluded that bad news about the conditions of the market inversely impacts the sociology as well as the psychology of investors. The highly pessimistic approach of media results in a negative impact on the market returns. According to the theory of investor sentiment, there is a consistent association between media content and the behavior of individual investors with extremely small stocks. This study established a new philosophy of investor psychology and the post-pandemic decision for investment. Only a few studies are there in the field; however, the majority of the studies focus on COVID-19 and human psychology as well as COVID-19 and the stock market. Investment decisions, as well as investors, are negatively influenced by the psychological pressure that may negatively impact the economy of an individual or country. This research attempts to investigate the psychology of investors and post-COVID-19 behavior of the stock market, which is a new debate in research comparatively. This work will contribute to the relevant literature in many ways. First, it will guide the exploration of new dimensions of investor emotions in relation to the investment decisions in the stock market more subjectively in the unusual circumstances of anxiety and pandemics. Next, this study will participate in the volume of studies associated with behavioral finance for future research reference. Then, new applications of Modern Portfolio Theory (MPT), Efficient Market Theory (EMH), Arbitrage Pricing Theory (APT), and Capital Asset Pricing Model (CAPM) are incorporated in this research that is quantitative theories and presumes perfect rational behavior of individual investors. After that, future researchers who are interested to undertake studies on the topic can also take help from this research. In addition, this is an important study for investors to develop their understanding of the significance of psychological elements concerning the decision-making of investors. Furthermore, the comprehensive background of the psychological factors and dynamic stock market variations will extend the understanding of students, investors, and scholars. Finally, this research will help investors making rational decisions by learning more about the association of psychological factors and the decision-making of individual investors because a better understanding will provide more confidence to the investors.

The article "Post-COVID-19 investor psychology and individual investment decision: A moderating role of information availability" was retracted in 2025. Reasons: unreliable results or conclusions; a conflict of interest; concerns about the peer review; concerns about the citations.

### Literature review

Social norms due to the pandemic’s severe effects and the potential threat of disease (Cao et al., 2020; Lai et al., 2020; Sarfraz et al., 2020). The anxiety, stress, and panic attacks of people due to COVID-19 have created two etiologies. The first is the identification of symptoms of acute respiratory distress syndrome (ARDS), such as cough and dyspnea, at high frequency (Javelot and Weiner, 2020). The second one is “false alarming” as a psychopathological link to the catastrophic interpretation of physiological sensation (respiration rate). The recurrence of panic attacks has increased the respiration rate and has become the reason for excessively avoidant behaviors and blind conformity (Li et al., 2020). Psychopathology is a keen concern for this study because it has an intense effect on investor’s behavior. Stock market investors and business people generally spend most of their time in the workplace. However, they are influenced human psychology through a notable mental state of “anxiety.” The term “anxiety” covers the population’s reaction toward the epidemic to all media, whether the information is authentic or erroneous, e.g., inappropriate behavior of people concerning the abandonment of animals and panic buying of other foods. The panic attacks are not properly defined without linkage to anxiety disorder in the medical sense. Anxiety is a combination of different psychiatric disorders, both internal (phobias, panic attacks, and panic disorder) and external (worry, stress, fear, painful experiences, or events). The psychological effect of COVID-19 has led to mass hysteria, post-traumatic stress disorder (PTSD), panic attacks, obsessive-compulsive disorder (OCD), and generalized anxiety disorder (GAD). The behavioral immune system (BIS) theory, stress theory, and perceived risk theory explain that negative emotion (anxiety and aversion) and negative cognitive assessment of human beings are developed for self-protection. People stock markets, investment decision pressure, and family members’ psychological health now put pressure on investor’s psychology. The COVID-19 outbreak has threatened every individual field of life to influence public health. The sustainability of the global stock market and financial markets also carries significant repercussions (Huang and Zheng, 2020). Being a part of the societal system, investor psychology (sentiments) and their optimism or pessimism about future stock prices can also change.

The article "Post-COVID-19 investor psychology and individual investment decision: A moderating role of information availability" was retracted in 2025. Reasons: unreliable results or conclusions; a conflict of interest; concerns about the peer review; concerns about the citations.

In the literature, a large number of researchers studied the consequences of calamities, including terrorism attacks, aircraft crashes, and earthquakes, on the financial decisions of investors and firms. Hassan and Hashmi (2015) conducted a study and concluded the very-short impact of terror attacks on the stock prices internationally, while this impact is more noticeable as compared to natural disasters, such as earthquakes.

In addition, Wang and Young (2020) determined that the risk aversion behavior of investors increases in response to terror attacks because these attacks create fear instead of something rational. Accordingly, Kaplanski and Levy (2014) found that in the case of aircraft crashes, the overreaction of investors is because of perceived risk increase instead of actual risk increase. The influence of the current COVID-19 epidemic is also acknowledged by the studies. Many researchers have the opinion that responses toward COVID-19 are shaped due to behavioral elements that include fear and uncertainty (Basheer et al., 2019). Illustratively, Gormsen and Koijen (2020) examined that the actual decrease in the prices of shares is higher than the expected decrease in growth because other elements are also influencing market conditions. Ramelli and Wagner (2020) found that level of the profits is too high to be controlled by the variations in cash flows instead of variations in discount rate because of uncertainty enhancement. Many other researchers concluded that previous experience with disasters, such as SARS, also influences market functioning. Ru et al. (2021) examined and found that economies with the experience of SARS face a fast decrease in market returns. However, Hassan et al. (2020) concluded that economies with the experience of SARS more positively deal with the COVID-19 situation. Hence, disasters and pandemics influence the understanding of people. The theory of behavioral finance depends upon the understanding of philosophy that in what ways emotions and cognitive biases shape individual investors’ behavior (Kengatharan and Kengatharan, 2014). In the field of behavioral finance, many of the scholars developed their studies based on cognitive psychology that deals with the thinking, reasoning, and decision-making of individuals or investors. Gitman et al. (2015) evaluate (Shannak and Obeidat, 2012). In addition, Bakar and Yi (2016) indicated that heuristics are commonly base on the exploration and application to find an appropriate solution to the issue. The behavioral finance model also incorporates conservatism and herding elements discussed by Kengatharan and Kengatharan (2014) and Wamae (2013) correspondingly. Previously, many studies have been conducted by scholars to evaluate the relation between psychological factors and the decision-making attitude of investors. More specifically, Ahmad Zaluki and Lim (2012) evaluated the association between psychological biases and the investor’s decision in the context of the Malaysian stock market. Here, psychological biases include “overconfidence bias, conservatism bias, herding bias, and regret bias.” He concluded the positive impact of overconfidence, conservatism, and regret concerning the decision-making of an individual investor. Conversely, an association of herding behavior was concluded to be neutral concerning the decision-making of an individual investor. The results of the study were majorly in line with the previous studies conducted in this context. In the Colombo stock market, Kengatharan and Kengatharan (2014) examined the association of behavioral elements with regard to the decisions of individuals. In addition, an association of behavioral elements and investment outcomes was also investigated. Kengatharan and Kengatharan (2014) concluded that herding, availability, and overconfidence bias in heuristics, prospect, and market elements are positively associated with individual investment decisions in Colombo Stock Market. Among these, most of the elements have moderate influences, excluding anchoring from heuristics that have a strong influence toward decision-making. In contrast, investment performance is influenced by only three of the evaluated variables. Herding factor variables and overconfidence from heuristics negatively affected investment outcomes. However, anchoring from heuristics has a positive influence on the performance of an investment. A positive association was found between the decision of investing with risk aversion, anchoring, prospect, and herding.

The article "Post-COVID-19 investor psychology and individual investment decision: A moderating role of information availability" was retracted in 2025. Reasons: unreliable results or conclusions; a conflict of interest; concerns about the peer review; concerns about the citations.

### Conceptual framework of the research model

In their book “Behavioral Finance,” Chandra and Thenmozhi (2017) presented key themes of behavioral finance that include “heuristics and biases, frame dependence, emotions, self-attributes, and inefficient markets”. Among these themes, some of the key psychological biases are incorporated in this study. These biases describe the main criteria that influence the decision-making of individual investors. A brief introduction of biases incorporated in this study is given below.

### Overconfidence bias

Cognitive bias refers to the individual’s overestimation of their capabilities, cognitive aptitudes, and accuracy of knowledge (Huisman et al., 2012) toward achieving their goals by disregarding or underrating future abnormalities. People with overconfidence assume that their observation s more correct as compared to that of others (Ahmad Sabir et al., 2019). They overreact to the information of the market (Broihanne et al., 2014). It is also concluded that male investors are more confident as compared to their female counterparts that leads them to an excessive transaction, which results in fewer profits (Abreu and Mendes, 2012; Broihanne et al., 2014; Metwally and Darwish, 2015). Moreover, Bessière and Elkemali (2014) evaluated overconfidence and self-attribution bias together and concluded that on the basis of personal knowledge, investors portray more confidence. Zaidi and Tauni (2012) also found that previous investment experience of investors affects their attitude in overconfident manners. Additionally, Mo et al. (2021) and Javed et al. (2017) found a positive association of overconfidence bias and the decision-making of the individual investor. However, their findings are dissimilar from the findings of Kengatharan and Kengatharan (2014), where they determined the negative association between variables. Therefore, the following hypothesis based on the extensive literature review is proposed.

**Hypothesis 1**: There is a significant association between overconfidence and investment decision of Chinese individual investors in the post-Covid-19 pandemic.

### Representative bias

Another name for this particular bias is “familiarity bias”. In the situation of lack of information or weak knowledge, neural processes use shortcuts to process this insufficient information to attain desired targets. Normally, information is evaluated on a previous experience basis. For instance, while purchasing a house, an individual will evaluate and compare prices of similar houses in that particular locality for understanding the property risk and future value of the asset. Representativeness refers to similar situations and occurrences in the population (Fama, 2021). Accordingly, Kahneman and Tversky (2013) have the opinion that usually people predict the future value of an asset-based on “representativeness.” This bias leads an investor to evaluate the characteristics of an organization that includes its executives, offerings, advertisement, and profits, and a general investment decision is made based on these components (Onsomu, 2014). In response to this bias, investors can make wrong decisions because of its focus on recent events where investors resultantly ignore long-term happenings (Shim et al., 2015). Investors with the representative bias neglect sample size and sometimes refer to very few samples (Jain et al., 2019). In addition, Alós-Ferrer and Hügelschäfer (2012) and Jha and Singh (2017) found this bias more prominent in inexperienced individuals. Javed et al. (2017) concluded that representative bias positively and significantly influences the perceived performance of an investment.

The article "Post-COVID-19 investor psychology and individual investment decision: A moderating role of information availability" was retracted in 2025. Reasons: unreliable results or conclusions; a conflict of interest; concerns about the peer review; concerns about the citations.

Therefore, the following hypothesis based on the extensive literature review is proposed.

**Hypothesis 2**: There is a significant association between representative bias and investment decisions of Chinese individual investors during the post-COVID-19 pandemic.

### Anchoring bias

This bias is concerned with the irrelevant comparison of stock price levels during the decision-making process. Investors with anchoring bias tentatively decide the price based on previous information while selling and buying shares. In this way, the timing of an investor’s decision may be wrong where he/she may sell stock at the time of decreased prices or may sell stocks at the time of increased prices. In addition, investors may lose good opportunities as their decided price for buying or selling may not be reached sometimes. This bias is also linked with the representative bias because the previous experience of investors is a common factor for both. Investors are commonly found optimistic about rising prices and are pessimistic about declining prices (Waweru et al., 2014). Investors rely on anchors while choosing an investment. Moreover, Jain et al. (2019) recommended in their research that anchoring methods are used by individuals while negotiating counteroffers, and by changing reference points, counteroffers are affected. Lee et al. (2013) added more than that anchoring bias is more common in women investors instead in men investors. Accordingly, Kengatharan and Kengatharan (2014) concluded that investors’ decisions are highly affected by the anchoring bias. Therefore, the following hypothesis on the basis of the extensive literature review is proposed.

**Hypothesis 3**: There is a significant association between anchoring bias and investment decisions of Chinese individual investors during the post-COVID-19 pandemic.

### Availability bias

Availability bias refers to the decision-making of an investor by relying on readily available information and ignoring other substitutes (Javed et al., 2017). When decisions are made based on recently happening events, decision-makers are perceived to portray availability bias. Personally experienced and observed recent happening are more unforgettable. For this reason, memorable happenings are tentatively more exaggerated, resulting in a demonstrative reaction. Moreover, investors decide their preferences in response to the available information even sometimes irrelevant information is also considered by them (Khan, 2017). Investors having this bias prefer to invest in local shares, which are commonly evaluated by professionals. Additionally, availability bias suggests that easily recalled events are perceived to happen with a greater likelihood (Rasheed et al., 2018). Institutional investor decisions are also affected by the availability bias (Siraji, 2019). Javed et al. (2017) concluded in their research that availability bias significantly and positively influences expected investment performance. In contrast, Khan (2017) and Rehan and Umer (2017) found that availability bias negatively influences decision-making regarding investment. The following hypothesis, based on an extensive literature review, is proposed.

The article "Post-COVID-19 investor psychology and individual investment decision: A moderating role of information availability" was retracted in 2025. Reasons: unreliable results or conclusions; a conflict of interest; concerns about the peer review; concerns about the citations.

**Hypothesis 4**: There is a significant association between availability bias and investment decisions of Chinese individual investors during the post-COVID-19 pandemic.

### Moderating role of availability of information

Literature on information searching endorses that the trading attitudes of investors are influenced by the accessibility of information. Similarly, studies of behavioral finance also concluded investment behaviors of individuals are influenced by their various cognitive skills. These deviations in investment behaviors need to be explained with new dimensions because they do not yet explain how information accessibility influences investment decisions in stock markets. Ahmad Sabir et al. (2018) surveyed accessing financial information and concluded that psychological factors, such as risk tolerance, cause changes in the information level of an individual by influencing information-gathering strategy. de Abreu et al. (2014) added that the accessibility of information provides the appropriate ground for decision-making regarding investment. Accordingly, investors who spent more time and money on information gathering can get summarized information on arising of investment opportunities and avail these opportunities more appropriately (Peress, 2014). In addition, Boyarchenko (2012) determined that quality information availability influences the attitude of investors; however, the reliability of available information is associated with the source of information. Investors make rational choices when they receive information from reliable sources (Guo, 2013). Furthermore, Bikas et al. (2013) have the opinion that while considering the opinion of financial experts, better self-assessment of investors is made on their own has a positive influence on the attitude of investors. Abreu and Mendes (2012) concluded significant positive relation between information accessibility and trading occurrence (Muneer et al., 1819). Tauni et al. (2015), in the context of China, confirmed the positive relation of acquiring information with behaviors of investors. By summing up, it seems that the psychological elements of an investor in decision-making are influenced by information availability. On the basis of the above literature review, these hypotheses are proposed.

The article "Post-COVID-19 investor psychology and individual investment decision: A moderating role of information availability" was retracted in 2025. Reasons: unreliable results or conclusions; a conflict of interest; concerns about the peer review; concerns about the citations.

**Hypothesis 5**: Information availability has a significant moderation role in the association of overconfidence with the investment decision of Chinese individual investors during the post-COVID-19 pandemic.

**Hypothesis 6**: Information availability has a significant moderation role in the association representative bias with the investment decision of Chinese individual investors during the post-COVID-19 pandemic.

**Hypothesis 7**: Information availability has a significant moderation role in the association anchoring bias with the investment decision of Chinese individual investors during the post-COVID-19 pandemic.

**Hypothesis 8**: Information availability has a significant moderation role on the association availability bias with the investment decision of Chinese individual investors during the post-COVID-19 pandemic.

## Research methodology

### Data collection method

The objective of this study is to investigate the influence of psychological biases on the investment decision of Chinese individual investors after the pandemic of COVID-19 with a moderating role of information availability. To attain the objective, a quantitative approach to research with a survey questionnaire is a suitable research technique (Kaur and Kaushik, 2016; Sabir et al., 2021). The survey questionnaire was planned with the supposition that it would be distributed among the individual investors of the stock market. Snowball sampling was used to collect the data. Chinese investors who are investing in the stock exchange were the population of the current study. A total of 400 survey questionnaires was disseminated among the target respondents. Out of 400 disseminated questionnaires, only 281 questionnaires were returned and able to use in the analysis. The response rate yield was 70.25%. The questionnaire was comprised of two sections. The first part comprises the questions demographics of respondents, while the second part consists of the items of investment decision, psychological biases information availability. A five-point “Likert scale” ranging from 1 “strongly disagrees” to 5 “strongly agree’ was applied to investment decision, psychological biases information availability. The Smart-PLS statistical software was employed to analyze the data and estimation of hypotheses. It is a software that uses the estimation of the relationships of all variables in a model simultaneously, and it is a second-generation technique to estimate the model (Hair et al., 2012, 2013). According to the suggestions of Hair et al. (2013), the method of bootstrapping with 300 resamples was applied for the estimation of hypotheses and path coefficients. This study follows the CFA method to check the validity of the model.

The article "Post-COVID-19 investor psychology and individual investment decision: A moderating role of information availability" was retracted in 2025. Reasons: unreliable results or conclusions; a conflict of interest; concerns about the peer review; concerns about the citations.

### Measurement model

Convergent validity (CV) and discriminant validity were investigated by using a measurement model. Convergent validity is used to estimate the degree that how different items measure the same concept. According to the suggestions of Hair et al. (2010, 2013), “factor loadings, composite reliability (CR) and average variance extracted (AVE)” are applied to assess CV. The suggested value for loading is 0.5, for AVE is 0.5 and for CR is 0.7. A measurement model is also used to examine the discriminant validity. Discriminant validity denotes the deviations among variables of the model. Discriminant validity is measured by the criteria of Fornell and Larcker (1981) and HTMT ratios. According to the criteria of Fornell and Larcker (1981), AVE’s square root should be greater than the correlations of that variable with others. Figure 1 below show the measurement model assessment.

**FIGURE 1:** Measurement model assessment.

In Table 1, convergent validity criteria are evaluated according to the recommendation of Hair et al. (2013) that meets the limit. Loading values were found larger than 0.6, CR larger than 0.7, and the AVE values found larger than 0.5.

**TABLE 1:** “Internal consistency, convergent validity, composite reliability, and average variance extracted (AVE)”.

Construct	Indicators	Loadings	Cronbach’s alpha	Composite reliability	AVE
Anchoring (AC)	AC1	0.813	0.889	0.924	0.752
	AC2	0.892			
	AC3	0.907			
	AC4	0.853			
Availability (AV)	AV1	0.698	0.843	0.885	0.608
	AV2	0.735			
	AV3	0.821			
	AV4	0.88			
	AV5	0.752			
Information availability (IA)	IA1	0.861	0.792	0.854	0.563
	IA2	0.857			
	IA3	0.774			
	IA4	0.682			
Investment decision (ID)	ID1	0.796	0.808	0.873	0.635
	ID2	0.800			
	ID3	0.792			
	ID4	0.759			
	ID5	0.768			
Overconfidence (OC)	OC1	0.873	0.947	0.959	0.824
	OC2	0.93			
	OC3	0.925			
	OC4	0.909			
	OC5	0.901			
Representative (RP)	RP1	0.825	0.813	0.877	0.642
	RP2	0.813			
	RP3	0.838			
	RP4	0.724			

In Table 2, discriminant validity criteria are assessed in line with Fornell and Larcker (1981) that also lies within the limit of achieving validity. All AVE square root values are larger than the correlations of respective variables.

The article "Post-COVID-19 investor psychology and individual investment decision: A moderating role of information availability" was retracted in 2025. Reasons: unreliable results or conclusions; a conflict of interest; concerns about the peer review; concerns about the citations.

**TABLE 2:** Fornell-Larcker criterion.

	AC	AV	IA	ID	OC	RP
AC	0.867					
AV	0.689	0.78				
IA	0.334	0.468	0.797			
ID	0.295	0.446	0.515	0.751		
OC	0.317	0.485	0.637	0.513	0.908	
RP	0.583	0.694	0.493	0.497	0.436	0.801

Table 3 represents that HTMT ratios that are smaller than 0.85. Hence, the research model meets the criteria of discriminant validity described by HTMT.

**TABLE 3:** Heterotrait–MONOTRAIT RATIO (HTMT).

	AC	AV	IA	ID	OC	RP
AC						
AV	0.792					
IA	0.387	0.549				
ID	0.4	0.521	0.607			
OC	0.349	0.534	0.732	0.575		
RP	0.684	0.796	0.596	0.581	0.496	

### Structural model evaluation

For the examination of the hypothesis, this research opted for the bootstrap method to test the association among independent, dependent, mediating, and moderating variables (Hair et al., 2013). The hypothesis was tested through bootstrapping of 1,000 resamples. Figure 2 below show the measurement model evaluation. Figure 2 and Tables 4, 5 demonstrate the findings of the structural framework.

**FIGURE 2:** Structural model assessment.

**TABLE 4:** Structural model assessment (direct effect results and decision).

Hypotheses	Relationship	Beta	STD	T value	*P*-values
**H1**	OC - > ID	0.295	0.078	3.782	0.011
**H2**	RP - > ID	0.342	0.062	5.516	0.016
**H3**	AC - > ID	0.214	0.072	2.972	0.017
**H4**	AV - > ID	–0.145	0.051	2.843	0.018

**TABLE 5:** Structural model assessment (moderation effects).

Hypotheses	Relationship	Beta	STD	T value	*P*-values
**H5**	OC*IA -> ID	0.178	0.043	4.139	0.011
**H6**	RP*IA -> ID	0.111	0.073	2.846	0.007
**H7**	AC *IA > ID	0.201	0.066	3.045	0.017
**H8**	AV*IA -> ID	0.109	0.043	2.534	0.015

*Relationship between variables.

Table 4 illuminates the results of the direct effects of psychological biases on investment decisions. Results illustrated that overconfidence significantly and positively influences to investment decision of Chinese individual investors (β = 0.0.295, *t* = 3.782) and representativeness bias also positively and significantly influences the investment decision of individual investors (β = 0.342, *t* = 5.516). Moreover, anchoring bias also has a significant influence on investment decisions (β = 0.214, *t* = 2.972). Furthermore, availability bias has a significant but negative influence on investment decisions (β = – 0.145, *t* = 2.843). Thus, H1, H2, H3, and H4 are supported.

The article "Post-COVID-19 investor psychology and individual investment decision: A moderating role of information availability" was retracted in 2025. Reasons: unreliable results or conclusions; a conflict of interest; concerns about the peer review; concerns about the citations.

Table 5 indicates the output of the moderation analysis. Results indicated that information availability significantly moderates the association of overconfidence, representative bias, anchoring bias, and availability bias with the investment decision of individual investors.

## Discussion

The first objective of this study was to investigate the decision after the COVID-19 outbreak among Chanies hypotheses of the study. This study found that on investment decision of Chanies individual investors significant and positive effect on investment decision (β = 0.342, *p* = 0.016). Anchoring bias also significantly influence on the investment decision (β = 0.214, *p* = 0.017). However, the availability bias has a significant but negative effect on the investment decision (β = –0.145, *p* = 0.018). These results are in line with the study of Sabir et al. (2019, 2021). Furthermore, information availability has a significant moderating role in the relationship among overconfidence, representative bias, anchoring bias, and individual investors, which is in line with the findings of Khan (2020).

## Conclusion

This study aimed to investigate the influence of psychological biases on the investment decision of individual investors after the COVID-19 pandemic. This study also intended to examine the role of information available on the relationship of psychological biases with the investment decision of individual investors. This a quantitative approach of research was employed to stock market. Results show that overconfidence, and positive influence on investment decisions; however, the availability bias has a significant but negative effect on the investment decision. Moreover, findings indicated that information availability has a significant moderating role in the relationship of psychological biases with the investment decision. The findings of the current study may benefit the participant of the stock market and other investors while they take the investment decision. The results of this study will contribute to the body of behavioral finance literature because it established the relevance of the prospect theory in illuminating the interaction between psychological factors, information availability, and the investment decisions of individual investors in a single model. Indirectly, this study offers a new direction in research on the predictors of investment decisions after the pandemic of COVID-19 in the context of China.

### Practical implications

This study will help financial specialists, economic institutions, and policymakers to generate better stock market strategies and make informed and rational investment decisions. This study also acknowledged the importance of various behaviors that has substantial impacts on investor investment decisions in the stock market during the post-COVID-19 pandemic. This study will assist such stock market experts and governments to know the importance of overconfidence, representativeness, anchoring, and availability biases in their investment decision. For making informed and rational investment decisions information availability for the investor is critical. However, effective legislation relating to information availability for investor is important to make significant investment decisions in the stock market. This study can also help us understand how information availability is important in identifying new investors who have not yet earned investment expertise and hence have not established investment strategy behavior during the post-COVID-19 pandemic.

The article "Post-COVID-19 investor psychology and individual investment decision: A moderating role of information availability" was retracted in 2025. Reasons: unreliable results or conclusions; a conflict of interest; concerns about the peer review; concerns about the citations.

### Limitations and future directions

Even though this study is unique in its proposition, there are limitations that should be addressed in future research. First, this study used a sample of Chinese investors. Thus, the results have limited generalized ability and changing the population in future research could validate the results of this study. Furthermore, this study has limited the four psychological biases that influence individual investors’ investment decisions.

Future research could investigate how the other psychological biases affect the investment decision of individual investors after the COVID-19 crisis.

## Data availability statement

The original contributions presented in this study are included in the article/supplementary material, further inquiries can be directed to the corresponding author.

## Ethics statement

Ethical review and approval was not required for the study on human participants in accordance with the local legislation and institutional requirements. Written informed consent from the patients/participants or patients/participants legal guardian/next of kin was not required to participate in this study in accordance with the national legislation and the institutional requirements.

## Author contributions

NJ presented the main idea, contributed to writing the original draft, and collected the data. JS contributed to the technique and methodology. KT performs the analysis. VJ revised and proofread the article. All authors contributed to the article and approved the submitted version.
